RETRACTED

# SNF5 promotes cell proliferation and immune evasion in non-small cell lung cancer

**DOI:** 10.1080/21655979.2022.2068894

**Published:** 2022-05-04

**Authors:** Ying Chen, Meilian Zhao, Dongliang Shen, Qian Yi, Liling Tang

**Affiliations:** a Key Laboratory of Biorheological Science and Technology, Ministry of Education, College of Bioengineering, Chongqing University, Chongqing, China; b Department of Physiology, School of Basic Medical Science, Southwest Medical University, Luzhou, China

**Keywords:** SNF5, NSCLC, proliferation, immune evasion, p-STAT3

## Abstract

Immune evasion is the process that tumor cells accelerate growth and metastasis by evading the recognition and attack of immune cells. SNF5 is one of the core subunits of SWI/SNF, which is involved in the development of a variety of malignancies. However, the functions of SNF5 in Non-Small Cell Lung Cancer (NSCLC) and the mechanism of SNF5 regulates immune evasion are still unclear. Based on this, we analyzed the expression of SNF5 and overall survival of lung cancer tissues through the cancer genome atlas (TCGA) database. Then we performed genetic gain and loss of function experiments with SNF5 using lentivirus infection and siRNA in NSCLC A549 and NCI-H1299 cells, respectively. We investigated the proliferation and immune evasion of these cells. We further explored the mechanism of SNF5 on NSCLC cells immune evasion. Our data showed that SNF5 was significantly increased in lung cancer tissues than that in normal lung tissues. Furthermore, SNF5 promoted NSCLC cells proliferation and the expressions of immune evasion-related genes. Meantime, overexpressed SNF5 reduced mortality of A549 cells when co-cultured with T cells. Moreover, SNF5 regulated the immune evasion by activating the signal transducer and activator of transcription (STAT3)/ phospho-STAT3 pathway in NSCLC cells. Together, our results validate SNF5 as a tumor oncogene and provide a new target for NSCLC treatment.

## Highlights

- SNF5 Promotes Cell Proliferation in NSCLC.
- SNF5 Promotes Immune Evasion in NSCLC.
- SNF5 regulated the immune evasion by activating STAT3/p-STAT3 pathway in NSCLC cells.

## 1. Introduction

Non-Small Cell Lung Cancer (NSCLC), one of the major types of lung cancer, has the highest mortality rate of all cancers [1]. Nowadays, therapeutic advances such as surgery, radiation therapy, chemotherapy, targeted therapies and immunotherapy, contributed to survival gains of NSCLC. However, the current status of NSCLC treatment is not optimistic due to treatment limitations, high postoperative recurrence rate, poor prognosis and low patient survival rate [2,3]. In addition, immune evasion is the hallmark of cancer and one of the major obstacles to increase the cure rate [4]. There are many reasons to induce the immune evasion of tumor cells, including the deficiency of costimulatory antigen on tumor cell, the reductions of killer immune cells, the increasing the number of immunosuppressive cells and the increasing the number of immunosuppressive factors in tumor microenvironment [5–7]. Therefore, it is necessary to explore the mechanism of immune evasion in NSCLC and find new therapeutic targets for NSCLC.

RETRACTED

Blocking immune checkpoint inhibitors, particularly the programmed cell death (PD-1)/ programmed cell death-ligand (PD-L1) signal, has enriched treatment strategies in NSCLC. PD-L1 and PD-L2 are the two major ligands PD-1. It is vital to explore the regulatory mechanism of PD-L1 to improve treatment in lung cancer. The repression of PD-L1 is regulated through several different ways in lung cancer. Previous studies have found that non-coding RNAs were involved in the translation of PD-L1. Hong et al. [8] found that let-7 miRNA binds to 3ʹuntranslated region (3ʹUTR) regions of PD-L1 and inhibits the expression of PD-L1 in NSCLC cells. In addition, Song et al. [9] also suggested that miR-138-5p has a bind site in 3ʹUTR regions of PD-L1. miR-138-5p, a tumor suppressor, inhibited tumor growth and immune evasion by down-regulating PD-L1 in NSCLC cells [10]. Furthermore, the cyclin-dependent kinase 7 (CDK7) is an oncogene in NSCLC. The inhibitor of CDK7 decreased the expression of PD-L1 by p38/MYC axis and increased CD8^+^ T cells infiltration. In addition, PD-L2, IDO1, TGF-β1 were also predictive biological maker of immune therapy efficacy [11–13].

SWI/SNF is a multi-subunit chromatin remodeling complex. The SWI/SNF ATPase subunit, BRG1 (also called SMARCA4), has been most studied in NSCLC. Xue et al. [14] suggested that loss of BRG1 decreased the expression of cyclin D1 and synthetic lethal with CDK4/6 inhibition in NSCLC. Moreover, loss of BRG1 also involved in activation of replication stress responses, cell growth, alteration of cellular morphology and increasement of tumorigenic potential in NSCLC [15–17]. And loss of SMARCE1 regulated the expression of epidermal growth factor receptor (EGFR) and resist mesenchymal-to-epithelial transition (MET) and anaplastic lymphoma kinase (ALK) inhibitors in NSCLC [18]. Sucrose Non-Fermenting Gene Number 5 (SNF5, also called SMARCB1, BAF47, INI1) was not inactivated in lung cancers and its functions were need to further confirmation [19]. Choi et al. [20] found that loss of SNF5 not only reduced cell cycle progression by upregulating p21 expression but also active immune response by upregulating IL-6 expression in human fetal lung fibroblasts IMR90 cells. The oncogenic functions of SNF5 were proved in recent research. They found that SNF5 was highly overexpressed in liver cancer patients and promoted cell proliferation, wound healing and tumor growth [21]. However, the functions of SNF5 in NSCLC were still unclear.

RETRACTED

In this study, we investigated the role of SNF5 in human NSCLC and found that the expression of SNF5 was up-regulated in human lung cancer tissues and was associated with poor prognosis. In addition, functional activation of SNF5 can promote the proliferation and immune evasion of NSCLC cells by activating STAT3/p-STAT3 signal pathway. Collectively, our results provide new insights into the role and molecular mechanism of SNF5 in NSCLC progression.

## 2. Materials and methods

### 2.1 Cell culture

The human NSCLC cell line A549 and NCI-H1299 were kindly provided by Dr. Yi Liao (The Southwest Hospital of AMU). A549 cell line was cultured in a F-12 K Medium (HyClone, USA) containing 10% fetal bovine serum (FBS), 100 U/ml penicillin, and 100 μg/ml streptomycin. NCI-H1299 cell line was cultured in a RPMI-1640 Medium (HyClone, USA) containing 10% FBS, 100 U/ml penicillin, and 100 μg/ml streptomycin. All cells were incubated in a humidified cell culture incubator with 5% CO2 at 37°C. All cell lines met the ethical requirements of Affiliated Chongqing University Cancer Hospital Ethics Committee (Ethical code: CZLS2022078-A).

### 2.2. Plasmids and siRNAs

Plenti-CMV-EGFP vector was purchased from Addgene. The Plenti-CMV-SNF5 vector was generated by adding SNF5 CDS regions to Plenti-CMV-EGFP instead EGFP position. These lentiviruses were produced in HEK293T using a mixture of lentivirus packaging plasmids (pCMV-dR8.2 dvpr and pCMV-VSV-G). The siRNA of SNF5 tar-get sequences designed by GenePharma (Shanghai) were the followings:

Negative scrambled siRNA: 5’-UUCUCCGAAGGUGUCACGUTT-3’

SNF5 siRNA: 5’- GUUGAUGACGCCUGAGAUGTT-3’

### 2.3. Reagents and primary antibodies

Polybrene and Puromycin were purchased from Sigma. The primary antibodies used in this study: SNF5(20,654-1-AP) and GAPDH (10,494-1-AP) were purchased from Proteintech. PD-L1(13,684), p21(2947), cyclin D1(55,506), STAT3(9139) and p-STAT3(9131) were purchased from Cell Signaling Technology. PD-L2 (ab187662) and IDO1(ab211017) were purchased from Abcam.

### 2.4. Quantitative real-time RT–PCR

RNA was extracted from cells using the RNAiso Plus kit (Takara Bio Inc.) and cDNA preparation was performed in accordance with manufacturer’s instructions using primeScript RT Master kit (Takara Bio Inc.). Real-time RT–qPCR was performed with SYBR qPCR SuperMix Plus (Annoronbio, China) using the 7300 Real-Time PCR System or ViiA7 System (AB Applied Biosystems). GAPDH was used as control. The primers used were as follows:

**Table:** 

	Forward (5′-3′)	Reverse (5′-3′)
GAPDH	AGAAGGCTGGGGCTCATTTG	AGGGGCCATCCACAGTCTTC
SNF5	GACGACGGCGAGTTCTAC	TCCTCTTGGCCTTCTGTT
PD-L2	ACCCTGGAATGCAACTTTGAC	AAGTGGCTCTTTCACGGTGTG
IDO1	TCTCATTTCGTGATGGAGACTGC	GTGTCCCGTTCTTGCATTTGC
PD-L1	TGGCATTTGCTGAACGCATTT	TGCAGCCAGGTCTAATTGTTTT
p21	CGATGGAACTTCGACTTTGTCA	GCACAAGGGTACAAGACAGTG
Cyclin D1	TGGAGCCCGTGAAAAAGAGC	TCTCCTTCATCTTAGAGGCCAC
TGF-β1	ATGGTGGAAACCCACAACGA	GCTGAGGTATCGCCAGGAAT

RETRACTED

### 2.5. Western blot

Cells were lyzed with RIPA buffer containing protease inhibitors cocktail and phosphatase inhibitor cocktail. Then the lysates were centrifugated at 12,000 rpm for 20 min at 4 C. The total protein concentration was measured by BCA protein assay kit (23,225, Thermo Fisher Scientific). Equal amounts of protein samples were separated by 10% SDS/PAGE and transferred to nitrocellulose membranes. After blocking with 5% milk, the membrane was incubated with the primary antibodies. After washing, the membranes were incubated with secondary antibodies. Signals were detected using the Bio-Rad gel documentation system with the Super Signal West Dura Extended Dura-tion Substrate (Bioscience, Shanghai).

### 2.6. Cell proliferation assay

At the indicated times (12, 24, 48 h and 72 h), A549 and NCI-H1299 cell lines were treated with CCK8 in 96 well plates, and the wells were incubated for an additional 1 h. Finally, Absorbance at 450 nm was evaluated using a Multiscan MS spectrophotometer.

### 2.7. T cell-mediated tumor cell killing assay

A549 and NCI-H1299 cells were co-cultured with CD3/CD28 T Cell Activator Cocktail and IL-2 pre-activated T cells sorted from human peripheral blood mononuclear cells for 24 h. The effector: target ratio was 1:1 or 5:1. The adherent cells were washed twice with PBS. Then CCK8 was added and the wells were incubated for an additional 1 h. The absorbance at 450 nm was measured and normalized to the absorbance of NSCLC cells incubated in the absence of T cells to obtain the percentage of viable cells.

### 2.8. ELISA assay

When T cells were activated with 100 ng/ml of CD3/CD28 and 10 ng/ml of IL-2 for 48 hours, the supernatant was collected and centrifuged at 1000 rpm for 10 min to remove the precipitate. According to the instruction of the ELISA kit (Jianglaibio, JL14556), the expression of IFN-γ in the cell culture medium was detected.

### 2.9. Statistical analyses

All statistical analyses were performed using GraphPad Prism6. The differences between the groups were compared by Student's t-test (comparing two variables) and one-way ANOVA analysis (comparing multiple variables). All data were presented as the means ±SD. Survival analysis was performed using the log-rank test. All p values < 0.05 were considered statistically significant.

RETRACTED

## 3. Results

In order to explore the mechanism of immune evasion in NSCLC and find new therapeutic targets for NSCLC, we firstly investigated the role of SNF5 in human NSCLC and found that the expression of SNF5 was up-regulated in human lung cancer tissues and was associated with poor prognosis. Then, we further found that SNF5 can promote the proliferation and immune evasion of NSCLC cells by activating STAT3/p-STAT3 signal pathway. Collectively, our results provide new insights into the role and molecular mechanism of SNF5 in NSCLC progression.

### 3.1. SNF5 was upregulated in human lung cancer tissues

To confirm the role of SNF5 in lung cancer, we first analyzed the mRNA level of SNF5 in human lung cancer patient tissues from the TCGA dataset. We found that the mRNA level of SNF5 is higher in human lung cancer patient tissues than in normal tissues (Figure 1(a)). Then we investigated the relationship between SNF5 expression and patient’s prognosis. Results showed that lung cancer patients with high SNF5 expression had a shorter overall survival than those with low SNF5 expression (Figure 1(b)). We further selected two additional different NSCLC sample databases, the Hou_2010 database containing 91 NSCLC samples and 65 adjacent normal lung tissue samples, the Baty_2010 database containing 29 chemotherapy-naive patients with NSCLC and 15 control patients with inflammatory lung diseases [22,23]. Further analysis of these two databases revealed that the expression of SNF5 is higher in human NSCLC tissues than in normal tissues and NSCLC patients with high SNF5 expression had a shorter overall survival than those with low SNF5 expression. These results indicated that SNF5 is a putative oncogene in lung cancer (Figure 1(c)-(f)).

**Figure 1.** SNF5 expression status in human lung cancer samples. a. In comparison with the SNF5 mRNA expression in non-tumor tissues(n = 59) and tumor tissue(n = 515) using TCGA database. b. The relation between the expression of SNF5 and the overall survival (OS) of lung cancer patients by database. c. In comparison with the SNF5 mRNA expression in non-tumor tissues(n = 65) and tumor tissue(n = 91) using Hou_2010 NSCLC database. d. The relation between the expression of SNF5 and the overall survival (OS) of NSCLC patients by database. e. In comparison with the SNF5 mRNA expression in non-tumor tissues(n = 15) and tumor tissue(n = 29) using Baty_2010 NSCLC database. f. The relation between the expression of SNF5 and the overall survival (OS) of NSCLC patients by database.

RETRACTED

By analyzing 29 NSCLC samples from the Baty_2010 database [23] (14 patients with high SNF5 expression and 15 with low expression), we showed that there was no significant association between high SNF5 expression and gender and age, that mortality was higher in patients with high SNF5 expression (60%) than in those with low expression (40%), and that SNF5 expression was associated with tumor grade (Table 1).

**Table 1.** Correlation of SNF5 expression and clinicopathological parameters in NSCLC patients

Variables	Total	SNF5		*P* value
		H	L	
Gender				
Male	19	8 (42.1%)	11 (57.9%)	0.599
Female	10	6 (60%)	4 (40%)	
Age(years)				
≥60	21	12 (57.1%)	9 (42.9%)	0.257
<60	8	2 (25%)	6 (75%)	
Death	15	9 (60%)	6 (40%)	0.052
Tumor grade				
I	6	3 (50%)	3 (50%)	0.023*
II	6	1 (16.7%)	5 (83.3%)	
III	6	6 (100%)	0 (0%)	
IV	11	4 (36.4%)	7 (63.6%)	

*p < 0.05.

### 3.2. SNF5 contributes to cell proliferation in NSCLC

First, we detected the expression of SNF5 in NSCLC cell lines A549 and NCI-H1299. The RT-qPCR results showed that the mRNA expression of SNF5 in the A549 cell lines was significantly decreased compared with the NCI-H1299 cell lines (Figure 2(a)). The same protein expression pattern was detected by western blots (Figure 2(b)). Then we overexpressed SNF5 in A549 cells and knocked down SNF5 in NCI-H1299 cells to explore the effect of SNF5 on the cell proliferation. A549-SNF5 cell line stably overexpressing SNF5 was constructed (Figure 2(c) and (d)). Then we detected the expression of proliferation associated proteins p21 and cyclin D1. Compared with the control A549-EGFP cells, overexpression of SNF5 down-regulated the expression of p21 and up-regulated the expression of cyclin D1(Figure 2(e) and (f)). CCK-8 assay showed that overexpression of SNF5 promoted the proliferation of A549 cells (Figure 2(g)). In addition, we designed siRNA to knock down SNF5 expression in NCI-H1299 cells. The RT-qPCR results and western blots results showed the expression of SNF5 decreased by SNF5-siRNA (Figure 2(h) and (i)). Compared to NCI-H1299 cells that transfected with nonspecific siRNA, inhibition of SNF5 expression increased the expression of p21 and decreased the expression of cyclin D1 (Figure 2(j) and (k)). CCK-8 assay showed that inhibition of SNF5 suppressed the proliferation of NCI-H1299 cells (Figure 2(l)). These results suggested that overexpression of SNF5 promoted the proliferation, while down-regulation of SNF5 inhibited the proliferation in NSCLC cells.

**Figure 2.** SNF5 contributes to cell proliferation in NSCLC. a. RT-qPCR analysis of the expression of SNF5 in A549 and H1299 cell lines. b. Western blot analysis of SNF5 expression in A549 and NCI-H1299 cell lines. c. RT-qPCR analysis statistics of the expression of SNF5 in A549-EGFP and A549-SNF5 cells. d. Western blot analysis of the expression of SNF5 in A549-EGFP and A549-SNF5 cells. e. RT-qPCR analysis of the expression of p21 and cyclin D1 in A549-EGFP and A549-SNF5 cells. f. Western blot analysis of the expression of p21 and cyclin D1 in A549-EGFP and A549-SNF5 cells. g. CCK8 assay analysis the proliferation of A549-EGFP and A549-SNF5 cells. h. RT-qPCR analysis statistics of the expression of SNF5 in H1299-NC and H1299-siSNF5 cells. i. Western blot analysis of the expression of SNF5 in H1299-NC and H1299-siSNF5 cells. j. RT-qPCR analysis statistics of the expression of p21 and cyclin D1 in H1299-NC and H1299-siSNF5 cells. k. Western blot analysis of the expression of p21 and cyclin D1 in H1299-NC and H1299-siSNF5 cells. l. CCK8 assay analysis the proliferation of H1299-NC and H1299-siSNF5 cells. (n = 3, *P < 0.05, **P < 0.01, ***P < 0.001).

RETRACTED

### 3.3. SNF5 acts as a modulator of immune evasion in NSCLC

As immune evasion is one of the important mechanisms in tumor progression, we explore the effect of SNF5 on immune evasion in NSCLC. Compared with the control A549-EGFP cells, overexpression of SNF5 upregulated the expression of immune evasion-related genes PD-L1, PD-L2, TGF-β1and IDO1 in A549 cells (Figure 3(a) and (b)). First, we tested the changes of IFN-gamma expression in T cells after stimulation by ELISA assay. The results showed that the level of IFN-gamma was significantly higher in antibody-stimulated T cells (Figure S1). Furthermore, CCK-8 assay showed that overexpressed SNF5 reduced mortality of A549 cells when co-cultured with T cells with ratio 1:1 or 5:1 (Figure 3(c)). Conversely, compared to NCI-H1299 cells that transfected with nonspecific siRNA, inhibition of SNF5 expression downregulated the expression of immune evasion-related genes PD-L1, PD-L2, TGF-β1and IDO1 (Figure 3(d) and (e)). Moreover, CCK-8 assay showed that deletion of SNF5 increased mortality of H1299 cells when co-cultured with T cells with ratio 1:1 or 5:1 (Figure 3(f)). In general, we hypothesis that SNF5 plays a promotion role in NSCLC immune evasion.

**Figure 3.** SNF5 plays an important role in regulating NSCLC immune escape. a. RT-qPCR analysis statistics of the expression of PD-L1, PD-L2, TGF-β1 and IDO1 in A549-EGFP and A549-SNF5 cells. b. Western blot analysis statistics of the expression of PD-L1, PD-L2, TGF-β1 and IDO1 in A549-EGFP and A549-SNF5 cells. c. CCK-8 assay analysis of A549-EGFP and A549-SNF5 cell lysis when co-cultured with T cells after 24 h with ratio 1:1(up) or 5:1(down). d. RT-qPCR analysis statistics of the expression of PD-L1, PD-L2, TGF-β1 and IDO1 in H1299-NC and H1299-siSNF5 cells. e. Western blot analysis statistics of the expression of PD-L1, PD-L2, TGF-β1 and IDO1 in H1299-NC and H1299-siSNF5 cells. Ff. CCK-8 assay analysis of H1299-NC and H1299-siSNF5 cell lysis when co-cultured with T cells after 24 h with ratio 1:1(up) or 5:1(down). (n = 3, *P < 0.05, **P < 0.01, ***P < 0.001).

RETRACTED

### 3.4. SNF5 regulates immune evasion through STAT3/p-STAT3 signaling pathway in NSCLC cells

To investigate possible mechanism of SNF5 regulated immune escape in NSCLC cell lines, we first detected the expression of p-STAT3 and STAT3. The phosphorylation level of STAT3 was higher in A549-SNF5 cells, while the phosphorylation level was decreased in NCI-H1299-siSNF5 cells (Figure 4(a) and (b)). As the above results showed, the STAT3 phosphorylation was correlated with SNF5 expression. To further confirmed whether p-STAT3 involved in regulation of immune evasion, we used a specific STAT3 inhibitor S3I-201 to inactivate STAT3 by blocking its phosphorylation and dimerization. S3I-201 was identified as an inhibitor of phosphorylation at Tyr-705 in the STAT3 transactivation domain and further inhibited the transcription of targe genes. Based on our data, the optimum concentration and processing time of S3I-201 was 150 µM and 24 h, which had no significant effect on the expression of STAT3 (Figure 4(c)). The presented data confirmed that the expression levels of PD-L2 and PD-L1 were increased in A549-SNF5 cells, while these increases were significantly reversed by S3I-201 administration, supporting SNF5 in promotion immune evasion by STAT3 pathway in A549 cells (Figure 4(d)).

**Figure 4.** SNF5 regulates immune escape through STAT3/p-STAT3 signaling pathway in NSCLC cells. a. Representative images show STAT3 and p-STAT3 protein expression in A549 cells that recombinantly express SNF5 or EGFP. b. Representative images show STAT3 and p-STAT3 protein expression in H1299-NC and H1299-siSNF5 cells. c. Screening the optimum treatment duration and concentration of S3I201. d. A549-EGFP and A549-SNF5 cells were treatment with S3I201(150 µm) or DMSO for 24 h. Protein expressions of p-STAT3, STAT3, PD-L2 and PD-L1 were detected by western blotting. (n = 3, *P < 0.05, **P < 0.01).

## 4. Discussion

SNF5, a core subunit of SWI/SNF, has been extensively studied in malignant rhabdoid tumors, pancreatic cancer and liver cancer [21,24,25]. Most researchers show that SNF5 is a tumor suppressor gene. However, in recent study, Hong et al. [21] found that SNF5 was upregulated in liver cancer patients and promoted cell proliferation, wound healing and tumor growth. These results suggested the oncogenic functions of SNF5. Consistent with these results, our research found that SNF5 was higher expression in lung cancer patients’ tissues than that in normal tissues and was associated with poor prognosis (Figure 1).

RETRACTED

Previous researches suggested that SWI/SNF play an important role in regulating tumor cell proliferation. For example, Zhou et al. [26] revealed that SMARCD1 promoted liver cancer growth via mTOR pathway. Wu et al. [27] found that BRG1 and BRM were overexpressed in triple negative breast cancers and promoted cell proliferation in vitro. Coincidentally, in SMARCD3-depleted breast cancer cells the proliferation rates were low and the expression of p21 was increased [28]. Our research added to this view and found that overexpression of SNF5 promoted NSCLC cells proliferation and regulate the expression of cell cycle-related protein (Figure 2).

Importantly, we further explored that SNF5 acts as a modulator of NSCLC immune evasion. On one hand, overexpression or knockdown of SNF5 in NSCLC cells altered the expressions of immune evasion related genes such as PD-L1, PD-L2, TGF-β1 and IDO1. On the other hand, overexpressed SNF5 reduced mortality of A549 cells when co-cultured with T cells. While deletion of SNF5 increased mortality of H1299 cells when co-cultured with T cells (Figure 3). Little research has been done on SNF5 in immunomodulation. Choi et al. [20] found that SNF5 bound with IL-6 prompter and inhibited IL-6 to prevent unnecessary immune responses. Our results complemented the role of SNF5 in the regulation of immunity and provided a new strategy for the treatment of NSCLC.

In nearly 50% of lung cancers, STAT3 can be activated by different upstream phosphokinases [29]. As a potential transcription factor, STAT3 in NSCLC has been shown to be involved in multiple processes including cell proliferation, differentiation, death and immune escape [30–33]. Researchers also found that STAT3 pathway regulated the expression of PD-1/PD-L1 and played antitumor immune response [34,35]. In addition, SWI/SNF and STAT3 pathway are closely related. Zhang et al. [36] found that SMARCA2 promoted pancreatic cancer growth and chemoresistance by activating STAT3 phosphorylation. Conversely, Wu et al. [37] suggested that STAT3 bound with the promoter of ARID1B and repressed the expression of ARID1B. We used S3I-201, an inhibitor of STAT3 phosphorylation, confirmed that SNF5 mediated the expression of immune-related genes with the involvement of p-STAT3 (Figure 4).

## 5. Conclusions

In summary, we found that SNF5, one of the core subunits of SWI/SNF, is an oncogene which is involved in the regulation of cell proliferation and immune evasion in NSCLC. These data enrich the mechanisms of SNF5-regulated immune evasion and provide a new insight for further understanding of immune evasion in NSCLC.

RETRACTED

## Supplementary Material

Supplemental Material
